# Predictive Value of Homeostasis Model Assessment of Insulin Resistance, Visceral Fat Index, and Prepregnancy Body Mass Index in Gestational Metabolic Syndrome

**DOI:** 10.1155/2021/6709725

**Published:** 2021-09-24

**Authors:** Laiping Zhao, Lichun Huang

**Affiliations:** ^**1**^ The Affiliated Nanhua Hospital, Department of Obstetrics and Gynecology Division 1, Hengyang Medical School, University of South China, Hengyang 421002, Hunan, China; ^2^The Affiliated Nanhua Hospital, Department of Joint Sports, Hengyang Medical School, University of South China, Hengyang 421001, Hunan, China

## Abstract

**Objective:**

To explore the diagnostic value of homeostasis model assessment of insulin resistance (HOMA-IR), visceral fat index (VAI), and prepregnancy body mass index (BMI) in gestational metabolic syndrome (GMS).

**Methods:**

From December 2019 to March 2021,122 GMS high-risk pregnant women who received routine antenatal clinic visits and planned to give birth in our hospital were selected as the research objects. Pregnant women were divided into the GMS group (*n* = 79) and the control group (*n* = 43) according to GMS diagnostic criteria during the gestation period of 32–36 weeks. The general information such as age and gestational week of pregnant women as well as HOMA-IR, VAI, and BMI before pregnancy were compared between the two groups. The glucose and lipid metabolism indexes of pregnant women in two groups were analyzed, the detection rates of HOMA-IR, VAI, and prepregnancy BMI in GMS between the two groups were compared. Logistic regression was used to analyze the risk factors for GMS in pregnant women, and receiver operating characteristic curve (ROC) was used to analyze the diagnostic value of HOMA-IR, VAI, prepregnancy BMI, and the combination of the three for GMS.

**Results:**

The body weight, systolic blood pressure, and diastolic blood pressure of the GMS group were higher than those of the control group, and the differences were statistically significant (*P* < 0.05). There was no significant difference in age, gestational week, and height between the two groups (*P* > 0.05). The levels of FPG, FINS, TC, TG, LDL-C, and FFA in the GMS group were higher than the control group, the level of HDL-C in the GMS group was lower than the control group, and the difference was statistically significant (*P* < 0.05). The levels of HOMA-IR, VAI, and prepregnancy BMI in the GMS group were higher than those in the control group, and the differences were statistically significant (*P* < 0.05). The positive detection rates of HOMA-IR, VAI, and prepregnancy BMI in the GMS group were 83.54%, 86.07%, and 81.01%, respectively. There was no significant difference in the positive detection rates of HOMA-IR, VAI, and prepregnancy BMI between the two groups (*P* > 0.05). High levels of HOMA-IR, VAI, and prepregnancy BMI were risk factors for GMS in pregnant women (*P* < 0.05). ROC curve showed area under the curve for HOMA-IR was 0.810, area under the curve for VAI was 0.771, and area under the curve for prepregnancy BMI was 0.749. The AUC for the combination of HOMA-IR, VAI, and prepregnancy BMI was 0.918.

**Conclusion:**

HOMA-IR, VAI, and prepregnancy BMI in GMS have a high detection rate and certain diagnostic value, and the combination of the three has higher clinical value.

## 1. Introduction

Gestational metabolic syndrome (GMS) is a group of syndromes occurring during pregnancy, which is mainly characterized by central obesity, insulin resistance (IR), abnormal metabolism of blood glucose and lipid, and other metabolic diseases [1, 2]. In recent years, with the improvement of living standards and changes in lifestyle, the incidence of GMS has increased significantly as compared with the past [3]. The pathogenesis of GMS is still unclear. Among them, IR is the central link in the occurrence and development of GMS [4, 5]. In order to meet the growth needs of the fetus, pregnant women will suffer from physiologically stressful IR, but excessive IR will lead to metabolic abnormalities of blood glucose and lipid, thus leading to the occurrence of GMS and increasing the risk of poor delivery outcome of pregnant women and poor prognosis of neonates [6, 7]. Homeostasis model assessment is clinically used to assess the insulin resistance index (HOMA-IR). HOMA-IR is an important indicator for assessing insulin sensitivity of patients and has a close relationship with insulin resistance, glucolipid metabolism disorder, and diabetes. Compared with single indexes such as waist circumference and weight, visceral obesity index (VAI) can be used to evaluate visceral fat dysfunction and cardiovascular risk factors. It can more accurately reflect the visceral fat content of patients and effectively predict the occurrence of GMS [8]. The prepregnancy body mass index (BMI) can be used to measure the nutritional status of the mother before pregnancy. The increase in prepregnancy BMI will increase the risk of GMS, which will lead to a significant increase in the incidence of neonatal weight abnormalities and adverse pregnancy outcomes [9, 10]. In this study, the levels of HOMA-IR, VAI, and prepregnancy BMI of pregnant women with GMS were observed and compared to analyze the risk factors for GMS in pregnant women and the diagnostic values of HOMA-IR, VAI, and prepregnancy BMI in GMS, so as to provide a practical basis for the clinical diagnosis and treatment of GMS. The specific report is as follows.

## 2. Data and Methods

### 2.1. General Information

From December 2019 to March 2021,122 GMS high-risk pregnant women who received routine antenatal clinic visits and planned to give birth in our hospital were selected as the research objects. The average age, height, and weight of 122 pregnant women were 28.01 ± 4.27 years, 161.05 ± 5.49 cm, and 63.32 ± 5.82 kg, respectively. Inclusion criteria: single pregnancy; patients with bad dietary habits such as sweet tooth; prepregnancy and abnormal weight during pregnancy; patients with previous adverse pregnancy outcomes and adverse pregnancy history; and complete clinical data. Exclusion criteria: patients with prepregnancy combined with metabolic syndrome; patients with severe abnormalities of cardiopulmonary function and liver and kidney function; infection during pregnancy; multiple pregnancy; late observation; and tracking cannot be completed according to the requirements of the research project. All pregnant women were grouped according to GMS diagnostic criteria from 32–36 weeks of gestation. Seventy-nine pregnant women diagnosed with GMS were included as the GMS group, and the remaining 43 pregnant women were included as the control group. This study was approved by the Ethics Committee of our hospital, and all patients or family members signed informed consent forms.

### 2.2. Research Methods

All pregnant women were measured for body weight, height, waist and hip circumference, blood pressure, blood glucose, and blood lipid during 9–13 weeks of gestation. Pregnant women take off their shoes and socks, wear light clothes, and measure their height and weight. When measuring the waist circumference, the pregnant woman takes the standing position, uses a tape measure with a spring ruler uniformly, and takes the middle point of the connecting line between the lower edge of the axillary midline rib arch and the iliac crest on both sides to read the value of the horizontal circumference. The blood pressure of the right upper arm in the resting state was measured by a desktop mercury sphygmomanometer for 2-3 consecutive times, and the average value of the results of the 3 measurements was taken. Fasting venous blood was collected in the morning, and the automatic biochemical analyzer was used to detect fasting plasma glucose (FPG), total cholesterol (TC), triglycerides (TG), and low density lipoprotein cholesterol (LDL-C), high density lipoprotein cholesterol (HDL-C), free fatty acid (FFA), and other biochemical indicators. Fasting insulin (FINS) was determined by radioimmunoassay.

Based on HOMA-IR = FPG (mmol/L) × FINS (mU/L)/22.5, HOMA-IR was calculated. Larger HOMA-IR value indicated more severe insulin resistance, and HOMA-IR ≥3.0 was positive. Based on VAI = (WHR/39.58+ (1.89 × BMI)) × (TG/0.81) × (1.52/HDL-C), in which BMI is kg/m^2^, TG and HDL-C are mmol/L. VAI was calculated as positive with VAI ≥3.8. The prepregnancy BMI of the pregnant woman was calculated based on BMI = weight/height^2^, and a positive prepregnancy BMI index of >25 kg/m^2^ was obtained.

Dynamic follow-up monitoring of the incidence of GMS in late pregnancy in all pregnant women and the diagnosis of pregnant women who met GMS criteria were performed. Diagnostic criteria of GMS: ① overweight or obesity before pregnancy, BMI >25 kg/m2; ② elevated blood glucose, diagnosed as gestational diabetes mellitus (GDM); ③ increased blood pressure, blood pressure ≥140/90 mmHg; ④ Abnormal lipid metabolism, TG ≥3.23 mmol/L/L. GMS can be diagnosed with three or all of these conditions [11].

### 2.3. Observation Indicators

The general information such as age and gestational week of pregnant women as well as HOMA-IR, VAI, and BMI before pregnancy were compared between the two groups. The glucose and lipid metabolism indexes of pregnant women in two groups were analyzed. The positive rates of HOMA-IR, VAI, and prepregnancy BMI in GMS were compared between the two groups to analyze the correlation between HOMA-IR, VAI, prepregnancy BMI and GMS components as well as its diagnostic value for GMS.

### 2.4. Statistical Methods

SPSS 20.0 software was used for processing. The measurement data of the experimental data were expressed as mean ± standard deviation, and the *t*-test was used for pairwise comparison. The count data were expressed as rate, and the comparison was performed using chi-square test. Receiver operating characteristic curve (ROC) curve was used to evaluate the diagnostic value. The test level was *α* = 0.05, and *P* < 0.05 indicated that the difference was statistically significant.

## 3. Results

### 3.1. Comparison of Clinical Data of Pregnant Women between the Two Groups

The body weight, systolic blood pressure, and diastolic blood pressure in the GMS group were higher than those in the control group, and the differences were statistically significant (*P* < 0.05). There was no significant difference in age, gestational week, and height between the two groups (*P* > 0.05) as shown in Table 1.

### 3.2. Comparison of Glucose and Lipid Metabolism Indexes between the Two Groups of Pregnant Women

The levels of FPG, FINS, TC, TG, LDL-C, and FFA in the GMS group were higher than the control group, the level of HDL-C was lower than the control group, and the difference was statistically significant (*P* < 0.05) as shown in Figure 1.

### 3.3. Comparison of HOMA-IR, VAI, and Prepregnancy BMI Levels in Pregnant Women between the Two Groups

The levels of HOMA-IR, VAI, and prepregnancy BMI in the GMS group were higher than those in the control group, and the differences were statistically significant (*P* < 0.05) as shown in Figure 2.

### 3.4. Comparison of the Positive Rates of GMS Detected by HOMA-IR, VAI, and Prepregnancy BMI in Pregnant Women between the Two Groups

The positive detection rates of HOMA-IR, VAI, and prepregnancy BMI in the GMS group were 83.54%, 86.07%, and 81.01%, respectively. There was no significant difference in the positive detection rates of HOMA-IR, VAI, and prepregnancy BMI between the two groups (*P* > 0.05) as shown in Figure 3.

### 3.5. Analysis of Influencing Factors of GMS in Pregnant Women

The occurrence of GMS in pregnant women was taken as the dependent variable, and age, gestational week, systolic and diastolic blood pressure, HOMA-IR, VAI, and prepregnancy BMI were taken as the independent variables, for multifactor logistic regression analysis.

The results showed that age, gestational week, and systolic and diastolic blood pressure were not influencing factors (*P* > 0.05), while high levels of HOMA-IR, VAI, and prepregnancy BMI were risk factors for GMS in pregnant women (*P* < 0.05) as shown in Table 2.

### 3.6. Diagnostic Value of HOMA-IR, VAI, and Prepregnancy BMI in GMS

ROC curve showed area under the curve for HOMA-IR was 0.810, area under the curve for VAI was 0.771, and area under the curve for prepregnancy BMI was 0.749. The AUC for the combination of HOMA-IR, VAI, and prepregnancy BMI was 0.918 as shown in Table 3 and Figure 4.

## 4. Discussion

For pregnant women, the body secretes a large amount of a variety of neuroendocrine hormones to meet the needs of fetal growth and development, resulting in long-term physiological emergency of pregnant women. When the secretion and regulation functions of hormones such as insulin and thyroid hormone are out of balance, it will cause metabolic diseases such as central obesity, hypertension, blood sugar, and blood lipid metabolism disorder [12, 13].

In recent years, with the growth of China's economic level, great changes have taken place in the national diet structure, which has led to an obvious increase in the incidence of metabolic syndrome. Guo et al.'s [14] research shows that the prevalence rate of metabolic syndrome in China is about 26.5%, especially in women. The physiological state of pregnancy, such as insulin resistance to a certain extent, accumulation of adipose tissue, and low-level inflammation of the whole body, can further promote its development towards metabolic syndrome, which together determines that the incidence of GMS is much higher than 26.5% [15]. GMS is one of the most common complications in obstetrics, and in severe pregnant women, it may induce complications such as premature birth, embryo loss, birth asphyxia, and fetal growth restriction, as well as adverse pregnancy outcomes [16]. GMS will also increase the risk of diabetes and cardiovascular disease in the long term. Therefore, in order to improve the adverse effects of pregnant outcomes and neonatal prognosis, early prediction is one of the important measures for effective prevention and control of GMS.

The GMS diagnostic criteria used in this study are objectively adjusted with reference to the diagnostic criteria of CDS metabolic syndrome and foreign research results [17]. Especially considering the physical characteristics of Chinese women, the BMI before pregnancy is generally lower than that of foreign women, and even obese women rarely exceed 30 kg/m^2^ before pregnancy. At the same time, the blood lipid level of pregnant women is physiologically upregulated. Therefore, BMI >25 kg/m^2^ and TG ≥3.23 mmol/L are more suitable for the physiological characteristics of Chinese pregnant women and can analyze the basic clinical characteristics of GMS more objectively.

In this study, there was no significant difference between GMS pregnant women and healthy pregnant women in terms of general information such as age and gestational age. However, the body weight, systolic blood pressure, and diastolic blood pressure in the GMS group were higher than those in healthy pregnant women, and the levels of FPG, FINS, TC, TG, LDL-C, FFA, and HDL-C in the GMS group were also significantly different from those in normal healthy pregnant women. Most pregnant women with GMS have increased BMI or obesity, increased blood glucose and blood pressure, abnormal lipid metabolism, etc., before pregnancy. Under normal conditions, a variety of hormones secreted by the placenta during pregnancy have a resistance effect on insulin and produce physiological IR, but a variety of inflammatory factors secreted by the obese pregnant women during pregnancy can lead to pathological IR [18]. Pathological IR refers to a state in which the sensitivity and reactivity of body tissues or target cells to insulin are decreased. The etiology is related to the dysfunction of insulin target tissues and insulin regulation disorder, which can lead to abnormal blood glucose and lipid metabolism, leading to the occurrence of GMS [19].

Obesity and insulin resistance jointly induce GMS under the influence of genetic factors, inflammation, and other factors [20, 21]. The results of this study showed that the levels of HOMA-IR, VAI, and prepregnancy BMI in the GMS group were higher than those in the control group. HOMA-IR is an effective indicator for easy estimation of insulin sensitivity, and the increase of HOMA-IR reflects the decrease of glucose handling ability and insulin sensitivity of pregnant women with GMS [22]. VAI, independent of gender, is an effective indicator of visceral fat dysfunction based on WC, BMI, TG, and HDL-C, suggesting increased visceral fat accumulation in GMS pregnant women [23]. In addition, the results of this study showed that the positive detection rates of HOMA-IR, VAI, and prepregnancy BMI in the GMS group were 83.54%, 86.07%, and 81.01%, respectively. However, there was no significant difference between the GMS pregnant women and the healthy pregnant women in HOMA-IR, VAI, and prepregnancy BMI positive detection rate. This is basically consistent with the research results of Jorquera [24] and Littlefield [25]. Clinically, prepregnancy BMI is often used to predict and evaluate the occurrence of GMS. However, due to the physiological IR in pregnant women during pregnancy, which leads to the compensatory increase of insulin, abnormal fat distribution, and excessive accumulation of visceral fat, prepregnancy BMI cannot completely predict the occurrence of GMS.

In this study, multivariate logistic regression analysis was used to analyze the related factors of GMS in pregnant women. The results showed that HOMA-IR, VAI, and prepregnancy BMI were the independent related factors of GMS in pregnant women. These results suggested that high levels of HOMA-IR, VAI, and prepregnancy BMI were risk factors for the development of GMS in pregnant women and might be used as potential diagnostic markers of GMS. In this study, the diagnostic values of HOMA-IR, VAI, and prepregnancy BMI for GMS were also analyzed by the ROC curve, which showed that the area under the curve of HOMA-IR was 0.810, that of VAI was 0.771, and that of prepregnancy BMI was 0.749. The AUC for the combination of HOMA-IR, VAI, and prepregnancy BMI was 0.918. This is basically consistent with the research results of Glueck [26] and Broughton [27]. These results indicated that HOMA-IR, VAI, and prepregnancy BMI had certain diagnostic value in GMS, and the combined diagnosis of the three factors was significantly improved compared with the single test, indicating that the combined diagnosis had higher clinical value. It can be used for early initial screening of pregnant women with GMS, which is conducive to early detection of GMS and preventive treatment.

There are still some limitations in this study: the number of cases is small, and the BMI level before pregnancy is affected by many factors. This study is only a cross-sectional study, and the significance of the results is limited. In the follow-up study, we should collect a large number of multicenter samples to further explore the mechanism of HOMA-IR, VAI, and BMI before pregnancy.

## 5. Conclusion

In summary, the levels of HOMA-IR, VAI, and prepregnancy BMI of pregnant women with GMS are significantly increased, which have a high detection rate and certain diagnostic value in GMS. In addition, the joint diagnosis of the three has higher clinical value and is a simple and effective indicator for early screening and preliminary diagnosis of GMS.

## Figures and Tables

**Figure 1:** Glucose and lipid metabolism indexes in pregnant women between the two groups. Note: compared with the control group, ^*∗*^*P* < 0.05.

**Figure 2:** HOMA-IR, VAI, and prepregnancy BMI levels in pregnant women between the two groups. Note: compared with the control group, ^*∗*^*P* < 0.05.

**Figure 3:** The positive rates of GMS detected by HOMA-IR, VAI, and prepregnancy BMI in pregnant women between the two groups.

**Figure 4:** ROC curve of HOMA-IR, VAI, and prepregnancy BMI in GMS.

**Table 1:** Comparison of clinical data between two groups of pregnant women (*n*, $\bar{x}$ ± s).

Group	Age (years)	Gestational week (week)	Height (cm)	Body weight (kg)	Systolic blood pressure (mmHg)	Diastolic blood pressure (mmHg)
Control group (*n* = 43)	28.04 ± 3.45	37.24 ± 1.79	161.47 ± 5.09	57.36 ± 4.18	114.64 ± 10.26	71.38 ± 10.57
GMS group (*n* = 79)	27.98 ± 4.27	37.18 ± 1.25	160.82 ± 4.72	66.57 ± 6.64	152.72 ± 14.83	92.64 ± 12.95
*t* value	0.079	0.217	0.706	8.241	14.986	9.218
*P* value	0.937	0.829	0.481	≤0.001	≤0.001	≤0.001

**Table 2:** Analysis of influencing factors of GMS in pregnant women.

Factor	B	Se	Wald's	*P*	OR	95% CI
Age	0.869	0.527	2.719	0.359	2.385	0.849–6.698
Gestational week	1.025	0.593	2.988	0.197	2.787	0.871–8.911
Systolic blood pressure	0.941	0.496	3.592	0.223	2.563	0.969–6.774
Diastolic blood pressure	0.982	0.604	2.643	0.208	2.669	0.817–8.721
HOMA-IR	0.579	0.219	6.989	0.011	1.784	1.162–2.741
VAI	0.692	0.317	4.765	0.019	2.001	1.073–3.718
Prepregnancy BMI	0.549	0.238	5.320	0.024	1.732	1.086–2.761

**Table 3:** Diagnostic value of HOMA-IR, VAI, and prepregnancy BMI in GMS.

Factor	AUC	S.E	95% CI	*P* value
HOMA-IR	0.810	0.040	0.731–0.889	≤0.001
VAI	0.771	0.047	0.679–0.864	≤0.001
Prepregnancy BMI	0.749	0.045	0.660–0.838	≤0.001
Combined diagnosis	0.918	0.033	0.854–0.983	≤0.001

## Data Availability

The data used during the current study are available from the corresponding author.

## References

[1] Rana S., Lemoine E., Granger P., Karumanchi S. A. (2020). Preeclampsia: pathophysiology, challenges, and perspectives. *Circulation Research*.

[2] Shen Y., Li W., Leng J. (2019). High risk of metabolic syndrome after delivery in pregnancies complicated by gestational diabetes. *Diabetes Research and Clinical Practice*.

[3] Hyer S., Balani J., Shehata H. (2018). Metformin in pregnancy: mechanisms and clinical applications. *International Journal of Molecular Sciences*.

[4] Samblas M., Milagro F. I., Martínez A. (2019). DNA methylation markers in obesity, metabolic syndrome, and weight loss. *Epigenetics*.

[5] Acton R. T., Barton J. C., Barton J. C. (2015). Serum ferritin, insulin resistance, and metabolic syndrome: clinical and laboratory associations in 769 non-hispanic whites without diabetes mellitus in the HEIRS study. *Metabolic Syndrome and Related Disorders*.

[6] Rogers J. M. (2019). Smoking and pregnancy: epigenetics and developmental origins of the metabolic syndrome. *Birth Defects Research*.

[7] Grieger J. A., Bianco-Miotto T., Grzeskowiak L. E. (2018). Metabolic syndrome in pregnancy and risk for adverse pregnancy outcomes: a prospective cohort of nulliparous women. *PLoS Medicine*.

[8] Srivastava R., Srivastava M., Verma P., Gautam A. (2019). Metabolic syndrome and periodontal disease: an overview for physicians. *Journal of Family Medicine and Primary Care*.

[9] Thong E. P., Codner E., Laven J. S. E., Teede H. (2020). Diabetes: a metabolic and reproductive disorder in women. *The Lancet Diabetes and Endocrinology*.

[10] Barquiel B., Herranz L., Hillman N., Burgos M. Á., Pallardo L. F. (2014). Prepregnancy body mass index and prenatal fasting glucose are effective predictors of early postpartum metabolic syndrome in Spanish mothers with gestational diabetes. *Metabolic Syndrome and Related Disorders*.

[11] Marciniak A., Patro-Małysza J., Kimber-Trojnar Ż., Marciniak B., Oleszczuk J., Leszczyńska-Gorzelak B. (2017). Fetal programming of the metabolic syndrome. *Taiwanese Journal of Obstetrics and Gynecology*.

[12] Iba T., Levy J. H., Levi M., Connors J. M., Thachil J. (2020). Coagulopathy of coronavirus disease 2019. *Critical Care Medicine*.

[13] Schnack L. L., Romani A. M. P. (2017). The metabolic syndrome and the relevance of nutrients for its onset. *Recent Patents on Biotechnology*.

[14] Guo H., Gao X., Ma R. (2017). Prevalence of metabolic syndrome and its associated factors among multi-ethnic adults in rural areas in xinjiang, China. *Scientific Reports*.

[15] Yao K., Bian C., Zhao X. (2017). Association of polycystic ovary syndrome with metabolic syndrome and gestational diabetes: aggravated complication of pregnancy. *Experimental and Therapeutic Medicine*.

[16] Heindel J. J., Blumberg B., Cave M. (2017). Metabolism disrupting chemicals and metabolic disorders. *Reproductive Toxicology*.

[17] Wiznitzer A., Mayer A., Novack V. (2009). Association of lipid levels during gestation with preeclampsia and gestational diabetes mellitus: a population-based study. *American Journal of Obstetrics and Gynecology*.

[18] Neuman H., Koren O. (2017). The pregnancy microbiome. *Intestinal Microbiome: Functional Aspects in Health and Disease*.

[19] Bhat M. A., Laway B. A., Shah Z. A., Wani A. I., Mubarik I. (2015). Insulin resistance, metabolic syndrome and chronic low grade inflammation in Sheehan’s syndrome on standard replacement therapy: a case control study. *Pituitary*.

[20] Noctor E., Crowe C., Carmody L. A. (2015). ATLANTIC-DIP: prevalence of metabolic syndrome and insulin resistance in women with previous gestational diabetes mellitus by International Association of Diabetes in Pregnancy Study Groups criteria. *Acta Diabetologica*.

[21] Neri C., Di Cesare C., Labianca A., Viggiano M., Caruso A., Paradisi G. (2018). Obesity in pregnancy as a model to identify women at risk for later metabolic syndrome. *Gynecological Endocrinology*.

[22] Ringholm L., Damm P., Mathiesen E. R. (2019). Improving pregnancy outcomes in women with diabetes mellitus: modern management. *Nature Reviews Endocrinology*.

[23] Klein A., Paradise L., Reeder M. (2018). Amenorrhea: a systematic approach to diagnosis and management. *American Family Physician*.

[24] Jorquera G., Echiburú B., Crisosto N., Sotomayor-Zárate R., Maliqueo M., Cruz G. (2020). Metformin during pregnancy: effects on offspring development and metabolic function. *Frontiers in Pharmacology*.

[25] Littlefield A., Lenahan C. (2019). Cholelithiasis: presentation and management. *Journal of Midwifery and Women’s Health*.

[26] Glueck C. J., Goldenberg N. (2019). Characteristics of obesity in polycystic ovary syndrome: etiology, treatment, and genetics. *Metabolism*.

[27] Broughton D. E., Moley K. H. (2017). Obesity and female infertility: potential mediators of obesity’s impact. *Fertility and Sterility*.

